The article "Intelligent Somatosensory Interactive Activities Restore Motor Function to Children with Autism" was retracted in 2023. Reasons: suspected computer-generated content; unreliable results or conclusions; lack of ethics approval or compliance; missing or withdrawn patient consent.

# Intelligent Somatosensory Interactive Activities Restore Motor Function to Children with Autism

**DOI:** 10.1155/2022/4516005

**Published:** 2022-03-27

**Authors:** Qiang Wang, Xing Wang, Lei Xu

**Affiliations:** ^1^School of Physical Education and Training, Shanghai University of Sport, Shanghai 200438, China; ^2^School of Sports and Health, Guangdong Polytechnic of Science and Technology, Zhuhai 519090, Guangdong, China; ^3^School of Physical Education, South China University of Technology, Guangzhou 510640, Guangdong, China

## Abstract

So far, the biomedical community has not provided clear etiological conclusions and targeted drug treatments. Educational intervention and rehabilitation are the main ways to promote the development of autistic children's ability and change the quality of life. This research mainly explores how intelligent somatosensory interactive activities can restore motor function to children with autism. Case studies are used to investigate the current problems of hand movement training for children with autism and the effect of somatosensory games on rehabilitation training for autism. The experience of autistic children using somatosensory games for hand movement training was analyzed. Through the collection, sorting, and analysis of data, the influence of different factors on users' immersive experience is explored. It designs and implements the system's somatosensory game module, including a detailed introduction to the development platform and key technologies used in the development of the somatosensory game module, and shows the functions, program flow, main features, and implementation effects of the somatosensory game. The development process of the somatosensory interaction system is introduced in detail, including model making, character control, task flow control, collision detection, interactive interface, and natural interaction methods of gesture interaction and voice interaction. This study outlines the concepts related to autism and the characteristics of children with autism. It discusses the feasibility of applying somatosensory games to the hand movement training of children with autism and analyzes the development status and application of somatosensory games in detail to lay the foundation for follow-up research. Moreover, it defines the research content of somatosensory interactive training products and clarifies the design content and direction of the product. The comfort evaluation of the somatosensory game products designed in the study reached 92.9%. This research further proves that somatosensory games have a positive effect.

## 1. Introduction

The specific injuries and external environmental factors of preschool children with autism reduce their chances of participating in physical activities, resulting in poor physical fitness. Social skills deficiency is one of the core defects of autism, which poses a lifelong challenge to autistic patients. However, the cause of autism is unknown, and it is a disease that accompanies life. So far, many medical experts have made unremitting efforts to relieve the symptoms of autistic patients, help them integrate into society, and improve their quality of life.

Mapping process for the study is as follows: In the first phase, therapists or teachers selected children with autism who met the inclusion criteria. In the second stage, the PEDI scale was used to evaluate the two groups of subjects, and the pretest data were obtained. The third stage is to accept the intervention of somatosensory games. In the fourth stage, after the children in the experimental group received the somatosensory game intervention, the posttest data were obtained. Active intervention training has an important role and value for autistic individuals, families, and society. First of all, active intervention can effectively reduce the degree of symptoms of autistic individuals; promote the development of various abilities such as language, social interaction, cognition, sports ability, and social adaptation; and lay a good foundation for survival and social life. Many autistic individuals can be greatly improved after active intervention training. During their adulthood, they can get jobs smoothly and become workers and creators of social wealth. This can bring good benefits to the society while reducing the cost of social welfare. This paper studies somatosensory interaction technology, applies natural human-computer interaction technology to training, and realizes the form of using computer technology to present training content. This paper realizes the interaction of multiple human senses and accurately distinguishes the participants in the training under the condition of interference. This achieves static gesture interaction and has achieved good practical results in application. At the same time, interactive gestures are used to replace most of the mouse operations. A desktop client for the cooperative ability training of children with autism spectrum disorder is realized. The use of sports games as an intervention can improve the motor ability of autistic children and can play a certain role in improving the daily behavior of autistic children. The purpose of this article is to design a more rigorous and scientific experimental plan based on previous research, to explore the effectiveness of somatosensory games in the intervention for children with autism, and to provide theoretical and data support for the application and promotion of somatosensory games.

## 2. Related Work

This paper uses the self-developed somatosensory game to intervene in children with autism and analyzes the effect of its intervention on the social skills, motor skills, and daily life skills of children with autism. After receiving intervention training, autistic individuals can return to society to participate in work. This not only can effectively reduce the cost of social welfare, but also provides the possibility of creating huge social benefits. Magnusson et al. believe that autism spectrum disorder (ASD) is a neurodevelopmental disorder. Its core characteristics are social communication barriers and atypical repetitive behaviors or restrictions on the scope of interest. These characteristics appear in the preschool stage and have a major and destructive effect in the subsequent developmental stage. It was able to reliably identify most cases well before the average age at diagnosis. This provides new opportunities for early intervention, but the availability of this intervention varies significantly among American communities, and its impact is not fully understood. Regarding the effectiveness of early enhancing behavioral interventions, there is a need for individualized therapy based on the genomic characteristics of individual patients. In addition, a new wave of research on the development of new therapies for newly elucidated causal effects will eventually change the clinical approach. These conditions occur in early childhood [1]. Salter and Stevens believe that a large number of new discoveries have recently given insight into the relationship between microglia and central nervous system (CNS) diseases. Understanding the physiological functions of these cells is essential to determine their role in disease [2]. Gandal et al. believe that the susceptibility of neuropsychiatric diseases involves a complex, polygenic, and pleiotropic genetic structure. However, little is known about how genetic variation can cause brain dysfunction or pathology. They use transcriptome analysis as a quantitative readout of molecular brain-based phenotypes for five major mental illnesses (autism, schizophrenia, bipolar disorder, depression, and alcoholism) and compare them with matched controls. This comprehensive system-level view of the neurobiological structure of major neuropsychiatric diseases shows ways of molecular convergence and specificity [3]. Lyall et al. believe that polychlorinated biphenyls (PCBs) and organochlorine pesticides (OCPs) are neurodevelopmental toxins, but few studies have examined the association with autism spectrum disorder (ASD). They aim to determine whether prenatal exposure to PCBs and OCPs affects the risk of ASD and nonautistic intellectual disability (ID) in offspring. They conduct a population-based case-control study in children born in Southern California. It includes children with ASD (*n* = 545) meeting the criteria of the Diagnostic and Statistical Manual of Mental Disorders 4th Edition (DSM-IV-TR) and ID (*n* = 181), as well as a general population (GP) control (*n* = 418). They compare the concentrations of 11 PCB homologues and 2 OCPs measured in stored serum samples of the second trimester between the diagnostic groups. Logistic regression is used to calculate the ratio (AOR) associated with ASD, and to calculate the ID, compared with the GP control, and the concentration of the primary research analyte [4]. Gilbert et al. believe that the understanding of the link between the human microbiome and diseases, including obesity, inflammatory bowel disease, arthritis, and autism, is rapidly expanding. The increase in throughput and accuracy of genomic DNA sequencing of microbial communities associated with human samples is supplemented by analysis of the transcriptome, proteome, metabolome, and immunome, as well as mechanical experiments in the model system. This greatly improves the ability to understand structure and function. However, there are still many challenges. In their comments, they focused on human research to describe these challenges and proposed using existing knowledge to quickly transform from correlation to causality and finally to a strategy that can be tried to solve the problem [5]. It can be found that the delay in the development of motor skills of children with autism is closely related to autism symptoms such as social communication disorders and repetitive stereotyped behaviors, emotional disorders, behavior disorders, and social adaptation skills. As the basis of the various fields, motor skills will play an important role in the overall development. Therefore, in the intervention in the fields of cognitive ability, language level, social communication skills, behavior, and emotion, it is also necessary to pay attention to the training of motor skills of children with autism. Somatosensory games intervention also has good effects on autistic children's daily living skills. In fact, educators already use somatosensory games in practice to improve skills related to daily living in children with autism.

## 3. Exploring Methods of Somatosensory Interactive Activities for the Recovery of Motor Function of Children with Autism

### 3.1. General Framework Design of Somatosensory Rehabilitation System

Kinect was used as a somatosensory interaction tool in this study. The system is divided into two modules in a targeted manner: somatosensory game module and data management module. The overall framework of the system is shown in Figure 1. The data management module of the system can view and manage game data on the server in real time.

### 3.2. Voice Interaction Module

Because Baidu Voice has the advantages of low user cost, support for multiplatform development, and diverse functions, it is used in this research to realize the voice interaction based on WorldViz. When using Baidu Voice's speech synthesis and speech recognition modules, you need to download and install the corresponding SDK package before development. Since Python is the development language in this research, only online speech synthesis Python SDK and online speech recognition Python SDK can be selected.

In games, dynamic sounds are more random, can reflect the interaction of various elements in the game, give players timely information feedback, and can better convey emotions. Although the dynamic sound will not change with the player's operation, it plays an important role in setting off and creating the atmosphere. Therefore, in game design, both dynamic sound and static sound play a very important role. In the design of somatosensory games, appropriate dynamic and static sounds should be selected according to the psychology of children with autism.

The spatial recognition degree is one-dimensional, and the direction of the sound source can be judged. However, accurate sound source localization cannot be carried out, and it needs to be combined with other auxiliary information to be able to proceed further [6].

(1) $$\begin{array}{c} d<\frac{\lambda }{1+\cos\;\phi }. \end{array}$$

*ϕ* is the incident direction of the sound source.

The far-field model needs to satisfy the distance *R* between the array and the loudspeaker [7].

(2) $$\begin{array}{c} R>\frac{\lambda L^{2}}{\phi }. \end{array}$$

Suppose the signal bandwidth is *B* and the array aperture is *L*; then, [8] one has the following:

(3) $$\begin{array}{c} \frac{L}{B}\leq 1. \end{array}$$

The signal model with reverberation can be modeled as follows:

(4) $$\begin{array}{c} y\left(t\right)=H\left(t\right)*S\left(t\right)+N\left(t\right). \end{array}$$

*S*(*t*) is the source signal.

The formula of array manifold vector is as follows [9]:

(5) $$\begin{array}{c} \alpha \left(z\right)=a\left(\beta ,\delta \right)=\left[\begin{array}{cc} e_{1} & e_{3}\\ e_{2} & e_{4} \end{array}\right],\\ z=-\frac{2\tau }{\lambda }\left[\begin{array}{cc} \sin\;\beta & \cos\;\varphi \\ \cos\;\varphi & \cos\;\beta \end{array}\right]. \end{array}$$

Among them, *z* is the wave number information of the sound source.

The parameters that need to be estimated in the sound source localization problem are *M* incident angle information [10].

(6) $$\begin{array}{c} y{\left(t\right)}_{L\times 1}=A{\left(\delta ,\varphi \right)}_{L\times M}S\left(t\right)+n{\left(t\right)}_{L\times 1},\\ A{\left(\delta ,\varphi \right)}_{L\times M}=\left[\begin{array}{ccccc} e^{-jz_{1}} & e^{-jz_{2}} & e^{-jz_{3}} & \ldots & e^{-jz_{n}} \end{array}\right]. \end{array}$$

The signal received by the microphone array can be modeled as follows:

(7) $$\begin{array}{c} y\left(t\right)=\left[y_{1},y_{2},y_{3},\ldots ,y_{n}\right],\\ y_{i}\left(t\right)=\sum_{m=1}^{M}y\left(t-\eta \right)+n\left(t\right),\\ \lambda ={\text{p}}^{T}\frac{v}{c}. \end{array}$$

Among them, *λ* is the time delay of *i* sound source relative to the origin and *m* microphone [11].

### 3.3. Database Logical Architecture

In the first layer, all network-based C/S network applications should include connection processing, authentication, and security management. The second layer is the core part of MySQL, usually called SQL Layer. The functions provided by each storage engine are concentrated in this layer, such as stored procedures, triggers, and views. The database items are shown in Table 1.

In the storage engine layer, the storage engine is really responsible for the storage and extraction of data in MySQL, and the server communicates with the storage engine through API. Different storage engines have different functions, so that we can choose the appropriate storage engine according to our own needs. Compared with other databases, MySQL is a bit different, and its architecture can be applied and played well in many different scenarios. Mainly reflected in the storage engine, the plug-in storage engine architecture separates query processing from other system tasks and from data storage and extraction. The third layer, storage engine, is usually called StorageEngineLayer. That is, the implementation part of the underlying data access operation. Storage engines cannot parse SQL, nor can they communicate with each other. They simply respond to server requests. The logical structure of the database is shown in Figure 2.

The objective function is defined as the weighted sum of four error squares [12]:

(8) $$\begin{array}{c} E=\gamma E+\gamma_{1}E_{S}+\gamma_{2}E_{N}B,\\ E_{D}={\underset{P\in T}{\sum }\left\|S\left(P\right)-D_{0}\left(P\right)\right\|}^{2}, \end{array}$$

where *E*_*D*_ is the distance between the estimated depth value *D*_0_(*P*) and the original depth value *S*(*P*) at the pixel point *p*.

Rectangular window [13] is as follows:

(9) $$\begin{array}{c} w\left(n\right)=\left\{\begin{array}{c} 1,\\ 0, \end{array}\right.\;\begin{array}{c} 0\leq n\leq m\\ else \end{array}. \end{array}$$

Hanning window is as follows:

(10) $$\begin{array}{c} w{\left(n\right)}_{\text{h}}=\frac{\left(1-\cos\;\delta /T\right)}{\gamma }. \end{array}$$

Gaussian window is as follows:

(11) $$\begin{array}{c} w{\left(n\right)}_{\text{g}}=e^{-\frac{1}{2}{\left(\alpha -\frac{n}{n-1}\right)}^{2}}=e^{-n^{2}/2\kappa }. \end{array}$$

*α* is the mean value [14].

### 3.4. Game Menu Design

The game menu interface of this system adopts Metro style design. Metro is the main interface display style of Microsoft Windows 8 operating system. It has the advantages of intuitiveness, simplicity, and strong maneuverability and is widely recognized by users. It makes the system interface more concise and intuitive and clear at a glance, with an excellent touch experience. In the control of the system interface, besides using traditional input devices such as mouse, keyboard, and touchpad, it also supports the function of human control. The system interface adopts the “hover selection” method to realize the human body's control of the system interface. When operating the system, the player only needs to move the palm to realize the menu selection function. There is a hand tool at the top of the system interface. When the player waves his/her hand to make a selection in the game menu, this hand tool will automatically track the position of the hand. Park your hand on the game you want to choose, and wait for the progress circle to fill up; then, the target game will be opened. This process will be completed within 2 seconds, and both left and right hands can realize the selection operation. It can get rid of traditional input devices, can easily control the system interface through the human body, and has a good control experience.

It represents its physical size in the physical coordinate system [15, 16].

(12) $$\begin{array}{c} \left[\begin{array}{c} u\\ v\\ 1 \end{array}\right]=\left[\begin{array}{ccc} \frac{1}{dx} & 0 & u\\ 0 & \frac{1}{dy} & v\\ 0 & 0 & 1 \end{array}\right]\left[\begin{array}{c} x\\ y\\ 1 \end{array}\right],\\ \left[\begin{array}{c} x\\ y\\ 1 \end{array}\right]=\frac{1}{\text{z}}\left[\begin{array}{ccc} f & -f\;\cot\;\varphi & 0\\ 0 & \frac{f}{\sin\;\theta } & 1\\ 0 & 0 & 0 \end{array}\right]\left[\begin{array}{c} x_{c}\\ y_{c}\\ z_{c} \end{array}\right]. \end{array}$$

Assumptions are as follows:

(13) $$\begin{array}{c} B=A^{-T}A^{-1},\\ H^{T}A^{-T}A^{-1}H_{2}=0. \end{array}$$

Therefore,

(14) $$\begin{array}{c} H_{1}^{T}A^{-T}A^{-1}H_{1}=H_{2}^{T}A^{-T}A^{-1}H_{2}. \end{array}$$

### 3.5. Children's Motor Function Coordination Test

#### 3.5.1. Leg-Eye Coordination Test Items

Leg-eye coordination is one of the branches of visual-limb movement coordination. The leg-eye coordination test project simulates catching a ball. The test requires sensitive and rapid lower limb movement ability, not only to quickly accelerate or decelerate the movement, but also to pay attention to the direction and position of the ball. At the same time, it is necessary to maintain the balance of the limbs during the movement. In the scene of the tested virtual playground, facing the Kinect camera, the computer automatically attaches the “bucket” to the tested body, and the movement of the “bucket” can be controlled by moving the body. Both yellow and green baseballs will drop on the top of the screen, and the test is conducted by moving the lower body to pick up the baseballs that fall from the air. This requires the tester to quickly move his/her lower limbs to catch the ball while observing the drop of the baseball above. At the same time, it must be adjusted according to the score and falling speed represented by the baseball to ensure that enough baseballs are received so that the final score will be higher. The final test result is based on the number of balls received in 1 minute.

(15) $$\begin{array}{c} P_{M}=P_{0}+P_{V}. \end{array}$$

*P*_0_ represents the position coordinates of the empty object, and its value is a fixed value, which can be set freely according to the specific situation; *P*_*V*_ is a random number.

(16) $$\begin{array}{c} V_{i}=V_{i-1}*0.9. \end{array}$$

*V*_*i*_ is the speed of the *i*-th ball [17].

#### 3.5.2. Hand-Eye Coordination Test

The project is based on conventional evaluation methods such as the 2-hand coordination test, double maze test method, sandbag throwing, and precision throwing, and it combines the characteristics of Kinect somatosensory interaction technology and the development characteristics of children's motor ability. The design idea of this test task is orbital push ball. This task aims to test the hand-eye coordination ability of children when they push the ball. In the 3D virtual high-altitude scene, children use four gestures to drive the ball forward, while preventing the ball from falling off the air orbit. There will be some “red gems” in the middle of the track. Children need to control the small balls to collect the “red gems” to increase the score. During this test, the computer automatically records the number of “red gems” collected. When children collect “red gems,” they need to convey the “red gems” they see to the brain and then control gestures to drive the ball to move to an accurate position. This is to control the speed of the ball and the displacement position of the ball. The more precise the children's gestures, the stronger the coordination and control ability of the muscles involved in sports, the higher the task completion, and correspondingly the higher their hand-eye coordination ability. If the child uses the wrong gesture during the operation, which causes the ball to fall off, the test is ended. The final test result is based on the number of “red gems” obtained without the ball falling. The lower right corner is the real-time three-dimensional animation of the human body, which can change according to the different movements of the human body. The testees can observe whether their movements are standard according to this picture.

#### 3.5.3. Auditory-Physical Movement Coordination Test Items

Auditory-limb movement coordination ability refers to the coordination of the response actions from the auditory organs to the corresponding body parts. According to the common test methods such as “follow the rhythm” and “change rhythm continuously,” the design idea of this task is to test the coordination ability of auditory-limb movement by “capturing the beat.” In the virtual scene, there are 5 color buttons, among which red, yellow, and blue are valid metronome, and the rest are invalid metronome. If you increase the difficulty of the test in the future, you can use the metronome of all 5 colors. The three-color metronome represents three different body movements, namely, raising the left hand, raising the right hand, and squatting. According to the prompts of the screen interface, the testee must maintain a high degree of attention and make corresponding physical movements in time to trigger the metronome. The distance of the different color beats on the screen is set according to the rhythm of the background music. Its perception of rhythm depends on the movement and hearing ability of the tested muscle system, as well as whether it can control the muscle movement in time when switching actions. If there is a rhythm error in the test process, it is often caused by the human muscles responding too fast or too slowly to the instructions of the brain. During the test, the computer automatically records the number of “metronomes” of different colors that are correctly triggered by the test. The test result is based on the correct number within a fixed time.

#### 3.5.4. Balance Test Items

Static balance ability test consists of the following: normal standing with eyes open, normal standing with eyes closed, standing on one foot, and standing on one foot with eyes closed. The dynamic balance ability test mainly records the score, the maximum angular velocity, the average angular velocity, the percentage of the time spent in the front, middle, rear, and left and right areas in the total test time of the testers, the time the ball stays in the center zone and zones 1, 2, 3, and 4, as well as the test score level. According to the existing test methods, such as “single-leg balance,” “jumping rope,” and “toe walking,” the “single-legged” task is designed. This project draws on the relevant indicators of the balance tester and the movement data of important bone points when the human body is standing on one foot. Hip Center is the key bone point of the human body when maintaining balance. The test indicators are as follows: the standing time on one foot, the total trajectory length of the skeletal point in the hip (Hip Center) within a fixed time, and the degree of shaking of the skeletal point [18].

(17) $$\begin{array}{c} LG=\sum_{i=1}^{n=1}\sqrt{{\left(x_{i}-x_{i-1}\right)}^{3}+{\left(y_{i}-y_{i-2}\right)}^{3}}. \end{array}$$

The formula is the converted two-dimensional position coordinates of the Hip Center collected by Kinect, and *n* is the number of collections. When the testee stands on one foot in the virtual test scene, Kinect will automatically recognize the one-foot standing action, start the test, and detect and identify the movement data of key bone points and the test time. If the tested feet touch the ground, the test automatically ends.

#### 3.5.5. Coordination Test between Limbs

During the test, the shorter the time it takes to complete the four movements, the better the coordination ability between the limbs. The test result is based on the correct number within a fixed time.

Assuming that *p*_*i*_(*f*), *p*_*i*_(*f*+1), *p*_*i*_(*f*+2) is the coordinate position data of the part for 3 consecutive frames, then the displacement vector is [19] as follows:

(18) $$\begin{array}{c} d_{i}\left(f\right)=p_{i}\left(f+1\right)-p_{i}\left(f\right),\\ d_{i}\left(f+1\right)=p_{i}\left(f+2\right)-p_{i}\left(f+1\right). \end{array}$$

Connect the Kinect power supply, make sure that the various lines are connected correctly, and start the Kinect hardware device. Obtain the status information of the device, and then let the children under test enter the visual range of Kinect (0.5–4.5 m). Kinect will detect the child's position and return the child's position parameters. At the same time, related applications began to calculate and draw the user's human skeleton image. In addition, it listens and constantly updates the skeleton image information. In order to prevent people from entering the test area by mistake and causing interference, Kinect will automatically detect the user closest to the device and ignore the undetected bone points [20].

## 4. The Result of Recovery of Motor Function in Children with Autism

The evaluation results of the two groups of ABC scales before the experiment are shown in Table 2. There is no significant difference (*p* > 0.05) in *S* (sensation ability), *R* (communication ability), *B* (motor ability), *L* (language ability), *S*2 (self-care), and total scores of the two groups before the experiment, and they are comparable.

There was no significant difference (*p* > 0.05) in the scores of the experimental group after treatment. The results of the significance evaluation of the experimental group after treatment are shown in Figure 3.

There was no significant difference in *S*, *R*, *B*, *L*, *S*2, and total score of the experimental group after the experiment (*p* > 0.05).  Table 3 shows the evaluation results of the ABC scale before and after the experiment in the control group.

The comparison results of the two groups of ABC scale evaluation scores before and after the experiment are shown in Figure 4. There is no significant difference (*p* > 0.05) in *S*, *R*, *B*, *L*, *S*2, and the total score between the two groups after the experiment.

The differences in perceived behaviors, gross movements, fine movements, language communication, cognitive behaviors, social behaviors, and self-care ability before and after training were statistically significant (*p* < 0.0001). The score comparison of various behaviors before and after training is shown in Table 4.

In cognition (*t* = 4.449, *p* < 0.0001), social (*t* = 3.914, *p* < 0.0001), and other aspects of the score difference before and after training, males are higher than females. This shows that the training effect on boys in these aspects is better than that on girls. The comparison of gender training effects is shown in Figure 5.

According to the classification criteria, the scores and total scores of 5 items are analyzed as shown in Table 5.

In order to give the subjects a more reasonable and targeted explanation, this article will analyze the test item scores of balance, hearing and limb coordination, limb coordination, hand-eye coordination, and leg-eye coordination, as shown in Table 6. The five test items are designed according to a certain element of the motor coordination ability, in order to explain the specific ability level of the subjects in a certain item. The scores of the 5 test items of the subjects were divided into 4 ability levels according to the standard deviation. We will analyze the 5 test items at different levels of progress at different ability levels.

It can be seen from Table 6 that in each project, there are 3 projects at ability level 1, and 2 projects at ability level 2. It can be seen from the results that most of the people with the first level of progress are at the level to be developed and the general middle level.

People at level 2 of progress are concentrated at level 2 of ability in each project. That is to say, most of the people at the second level of progress are at the general middle level. The ability level analysis is shown in Figure 6.

Pediatric Evaluation of Disability Inventory (PEDI) is a professional scale for functional assessment of children with low abilities. It can effectively detect the impairment of each field or energy area of children with disabilities, judge the efficacy of rehabilitation, formulate rehabilitation plans, and guide rehabilitation training. Statistical analysis of the data was performed, and the analysis results are shown in Figure 7. The scores of PEDI scale of daily living ability improved more obviously.

According to the weight ranking of evaluation indicators, in the interaction design of somatosensory games, the evaluation indicators have the largest weight. This shows that the evaluation index is more important and should be given priority in the design. The ranking of evaluation indicators is shown in Figure 8.

It can be seen from Figure 8 that the simple screen, simple operation, and straightforward interface level in the evaluation index account for a larger weight. In order to save the cost of design, these indicators should be given priority in the design.

A total of 28 people participated in the design evaluation, including 10 teachers and 18 parents. 28 questionnaires were returned, of which 28 were valid questionnaires. 92.9% of people think that the training process can meet the requirements of comfort, 89.3% of people think that training aids can bring a positive experience to the training of autistic children, 100% of people think that the design plan meets the requirements of function, and 96.4% of people think that the design can achieve the desired effect and improve the user experience of the training process. The evaluation result of the system is shown in Figure 9.

## 5. Discussion

The structural characteristics of children with autism determine their functional status, and dysfunction affects their normal growth and development mode, which ultimately leads to structural changes. Social communication barriers restrict the reception and feedback of external information in children with autism, and repetitive stereotyped behaviors restrict the development of complex continuous movements in children with autism [21].

Appropriate sports participation will have a positive impact on children's basic sports ability, quality of life, healthy lifestyle, emotions, and psychology. However, because children with autism are closed in their own world, they are unwilling to receive information from the outside world or even resistant to this. As an effective internal stimulating factor, sports are not easy to reject by children with autism, and sports can provide opportunities to increase the interaction and communication behavior of children with autism [22].

Exercise can enhance and is beneficial to physical and mental health, and cognitive and intellectual development. For example, activities such as hand-slapped basketball and foot-passing football improve children's hand-eye coordination and visual concentration; running and frog jumping on the road improve the coordination and flexibility of children's limbs and torso; and lifting small dumbbells, squatting, jumping, and frog jumping can increase the muscle strength of children's limbs, which is of great help to the improvement of physical coordination. Jogging can exercise children's endurance, and cardiopulmonary function can also be improved. The practice of abdominal breathing and blowing games can adjust the breathing pattern of children with autism and improve cardiopulmonary function. Repeated practice of all aspects of movement in sports can not only promote the improvement of athletic ability and lay a good foundation for the later development of motor skills, but also exercise self-control.

In order to better serve children with autism and let the rehabilitation of children with autism embark on a path of sustainable development, it is necessary to increase the rehabilitation staff and management team with rich experience and strong professional ability. Corresponding measures should be taken to stabilize the professional team of rehabilitation personnel and prevent the loss of employees. Rehabilitation personnel responsible for children with autism improve their rehabilitation skills and actively adjust their mentality through continuous learning. They accept short-term rehabilitation training for children with autism implemented by the Disabled Persons' Federation and other departments, learn the most cutting-edge rehabilitation skills in the field of children's autism rehabilitation, and skillfully apply them in rehabilitation work. Rehabilitation institutions check when personnel are admitted, recruit high-quality personnel based on the core competence requirements of child autism rehabilitation personnel, guide and promote the self-development of rehabilitation personnel through the assessment and review system, and improve the capabilities of rehabilitation personnel through the provision of systematic on-the-job training and academic exchanges.

To a certain extent, autism is a specific behavioral disorder and excessive syndrome, with the inability to carry out normal social activities like ordinary children. Therefore, it is particularly important to take effective and scientific interventions for stereotyped behaviors. There are many similarities between sensory integration disorder and stereotyped behavior in behavior performance, which is easy to cause confusion. Therefore, scholars who pay attention to this field explore the relationship between the two and come to the conclusion in the process of exploring the reasons for the occurrence of stereotyped behavior: the main internal reason for the occurrence of stereotyped behavior is to seek sensory stimulation [23].

In recent years, although the society as a whole has continuously deepened the understanding of autism, there is still a certain gap between the research on social support, social welfare, and security system of autistic children and foreign countries. Personnel engaged in education in special schools also urgently need a set of methods that have proven effective through theoretical and practical research to educate children with autism.

Often, many children with autism will show a clear sense of anxiety, and they will unconsciously relieve their anxiety through various stereotyped behaviors. This situation will cause children to be in an idle state, which will show stereotyped behaviors to seek various stimuli. Therefore, it is particularly important to seek professional treatment organizations to arrange reasonable treatment plans for children with autism and to provide children with a relaxing and pleasant treatment environment. In addition, parents can scientifically and rationally arrange their children's treatment plan with the teacher, improve the efficiency of rehabilitation, and develop scientific and reasonable living habits [24].

The description and evaluation of the functional status of children with autism should be carried out by professionals. The functional status of children is a process of dynamic balance between the individual and the environment. In the evaluation, the child's family situation and the situation of the school or rehabilitation institution should also be fully considered. Rehabilitation training for children with autism is a long process and requires more care and support from the family and society. Therefore, a family-school or rehabilitation institution-society long-term close cooperation relationship should be established to jointly create a good rehabilitation training and living and learning environment for children with autism [25].

## 6. Conclusion

Studies have shown that somatosensory games are effective in rehabilitation training for children with autism. However, it is rare to design a somatosensory game based on the characteristics of autistic children from the perspective of interaction design and user experience design to enhance the initiative and enthusiasm of the training of children with autism, thereby improving the effect of training. Through the design and implementation of the experimental program, the subjects are trained in a planned way, and the effectiveness of the system is finally verified by analyzing the training data and evaluation data of the subjects. The use of advanced computer technology to partially replace the traditional training model also provides a certain reference. However, this study found that there are many problems in the use of somatosensory games for hand training in children with autism after field investigation, and training aids must be used to achieve the best results. This requires research on the form and function of training aids to improve the user experience of autistic children during training. Therefore, this research has great research prospects. Healthcare intervention based on intelligent interactive gesture technology can scientifically and effectively exercise the muscle strength and balance, throwing, jumping, and climbing abilities of children with autism; visual responses, anxiety responses, verbal communication, and interpersonal relationships were improved. Somatosensory games can effectively stimulate the learning motivation of children with autism and show good intervention effects. Therefore, in the intervention practice of children with autism, it is possible to appropriately combine somatosensory games on the basis of existing intervention methods to intervene in children with autism, to improve the intervention effect for children with autism.

## Figures and Tables

**Figure 1:** The overall framework of the system.

**Figure 2:** Database logical architecture.

**Figure 3:** Significance evaluation results after treatment in the experimental group.

**Figure 4:** Comparison between the two groups of ABC scale evaluation scores before and after the experiment.

**Figure 5:** Comparison of gender training effects.

**Figure 6:** Ability level analysis.

**Figure 7:** PEDI scale score.

**Figure 8:** Ranking of evaluation indicators.

**Figure 9:** Evaluation results of the system.

**Table 1:** Database items.

Field name	Type	Field description
Pro name	Varchar (32)	Project name
Pro code	Varchar (20)	Project code
Type	Varchar (20)	Project type
Researcher	Varchar (20)	Project contributor

**Table 2:** Evaluation results of the two groups of ABC scales before the experiment.

Subscale parameters	Experimental group (*n* = 18)	Control group (*n* = 14)	*P*
*S* (sensory ability)	9.83 ± 7.326	10.428 ± 5.543	0.802
*R* (communication ability)	10.889 ± 8.858	11.57 ± 7.165	0.816
*B* (exercise ability)	6.556 ± 6.401	8.36 ± 7.239	0.461
*L* (language ability)	12.833 ± 7.422	8.79 ± 7.106	0.130
*S*2 (self-care)	9.556 ± 6.061	8.57 ± 3.715	0.598

**Table 3:** Evaluation results of the ABC scale before and after the control group experiment.

Subscale parameters	Before the experiment	After the experiment	*P*
*S* (sensory ability)	10. 428 ± 5.543	11. 571 ± 5.867	0.680
*R* (communication ability)	11.57 ± 7.165	12.357 ± 6.368	0.396
*B* (exercise ability)	8.36 ± 7.239	11.214 ± 7.392	0.929
*L* (language ability)	8.79 ± 7.106	11. 142 ± 8.11	0.114
*S*2 (self-care)	8.57 ± 3.715	10.928 ± 4.322	0.625

**Table 4:** Comparison of scores of various behaviors before and after training.

Subscale parameters	Before training	After training	Score difference before and after training
Perceptual behavior	23.76 ± 0.94	39.07 ± 0.99	15.31 ± 0.80
Gross movement	36.63 ± 1.21	55.71 ± 1.10	19.08 ± 0.79
Fine motor	31.64 ± 1.30	46.21 ± 1.18	14.57 ± 0.62
Language communication	25.03 ± 1.63	48.01 ± 1.64	22.98 ± 1.11
Cognitive behavior	17.64 ± 1.03	34.82 ± 1.18	17.18 ± 0.87
Social behavior	17.38 ± 0.74	30.85 ± 0.84	13.48 ± 0.65

**Table 5:** Analysis of the scores and total scores of 5 items according to the classification criteria.

Project	Progress level one	Progress level two	Progress level three	Progress level four
Balance test	4	13	18	4
Auditory-physical coordination test	4	15	15	5
Limb coordination test	4	10	20	3
Hand-eye coordination test	5	14	17	4
Leg-eye coordination test	5	12	18	4
Total score	1	18	18	2

**Table 6:** Detailed analysis of the test item scores of balance, auditory-limb coordination, limb-limb coordination, hand-eye coordination, and leg-eye coordination.

Project	Progress level 1	Progress level 2	Progress level 3	Progress level 4
Balance test	1	0	0	0
Auditory-physical coordination test	1	0	0	0
Limb coordination test	1	0	1	0
Hand-eye coordination test	0	0	0	0
Leg-eye coordination test	0	1	0	1

## Data Availability

No data were used to support this study.
